The article "Application of Biomechanics Based on Intelligent Technology and Big Data in Physical Fitness Training of Athletes" was retracted in 2023. Reasons: unreliable results or conclusions; concerns about the data; concerns about the peer review; concerns about the citations.

# Application of Biomechanics Based on Intelligent Technology and Big Data in Physical Fitness Training of Athletes

**DOI:** 10.1155/2022/7323146

**Published:** 2022-08-26

**Authors:** Kai Li, Jinqian Zhang, Qingling Qu, Bairan Li, Sukwon Kim

**Affiliations:** ^1^Department of Physical Education, Jeonbuk National University, Jeonju 54896, Jeollabuk, Republic of Korea; ^2^College of Physical Education, Pingdingshan University, Pingdingshan 467000, Henan, China

## Abstract

Physical training has a high degree of participation all over the world. With the opening of the era of national fitness, physical training has become more popular from the original specialization, and the complex training methods and contents have gradually become simplified. The development and change of physical training has also brought many problems to the professional training of athletes, such as high training intensity but poor effect, insufficient training posture, and long-term physical injury. In order to help athletes achieve better results in physical training and reduce the probability of injury, taking sprint training as an example, this article adopted the sports and body data of elite athletes through intelligent technology and big data analysis, established a human motion model from the perspective of biomechanics, and then conducted a corresponding test run experiment for athletes. The experimental results suggested that drag resistance running could improve the specific strength quality of sprinting. At the same time, when using resistance load for training, the maximum speed should not exceed 90% of the maximum speed without resistance. The average horizontal maximum velocity decreased by approximately 9% when training under a resistance load, and the best training results were obtained by training athletes within this range.

## 1. Introduction

Physical training is an important factor in improving athletes' specific performance and competitive ability. How to improve athletes' performance and reduce injury rates in physical training has always been a hot topic in the sports world. The traditional research method is to let athletes perform repeated exercises through various physical training methods, but this method has the risks of uncertain training results and high training injury rate. With the advent of the digital age, big data has become a powerful tool for analyzing and comparing dense data, and big data analysis has provided a lot of digital support for physical training. Big data can collect key information about athletes' bodies before and after training and digitize them in combination with corresponding physical training to apply them to training to improve athletes' performance. At the same time, a large number of athletes' physical and training information can be collected to guide the corresponding sports training. However, the amount of data required for this work is too large, which brings many challenges for training reference. At present, there are few studies on digital physical training in the academic field, mainly focusing on the application of modern intelligent sports equipment and data analysis of athletes' training and competition.

The article "Application of Biomechanics Based on Intelligent Technology and Big Data in Physical Fitness Training of Athletes" was retracted in 2023. Reasons: unreliable results or conclusions; concerns about the data; concerns about the peer review; concerns about the citations.

In addition to the data analysis brought by the digital age, the study of biomechanics also provides good guidance for physical training. Biomechanics is a branch of biophysics that uses the principles of mechanics to quantitatively study mechanical problems in living organisms. Biomechanics can analyze the force of key parts in the process of athlete's movement and training, evaluate the training effect of the athlete, and provide a safety reference for the athlete's training to avoid injury. In the era of “big data,” the collection, analysis, evaluation, and feedback of relevant data in the training process of athletes have become an important means to improve training effectiveness. Intelligent big data analyzes the skills and physical conditions of athletes and can combine biomechanics to improve athletes' training to achieve good training results. The innovation of this article is that it simplifies the amount of intelligent big data analysis without affecting the research results. From a biomechanical point of view, starting from sprinting, a popular but very scientific sport, after collecting information on athletes, a unique human model was constructed to evaluate the performance of comparative athletes, resulting in good experimental results.

## 2. Related Works

With the continuous development of competitive sports, the frequency of various sports meetings and sports events is increasing day by day, physical training is no longer the patent of athletes, and the research on physical training has also expanded to all aspects of daily life. Grier studied the effects of physical training and fitness on running injuries in physically active young men and found that a greater risk of running injuries was associated with older age, higher BMI, and total running distance per person [1]. This research could help people exercise more safely, but the findings were still too broad and not specific. Chainay started from the elderly in the research of physical training and proposed that good physical training could effectively improve the cognitive ability of the elderly [2]. Although his research is helpful for physical training in the elderly, it does not provide a good risk control. However, it is unclear whether the combination of cognitive and physical training has advantages over cognitive training alone. Bartnovskay focused on the field of women's physical training, formulated health-related application techniques for special healthy women (with health problems), and evaluated its impact on physical conditions [3]. This study broadened the target population of physical training and also provided good assistance to female athletes. The scope of his research is too small, so further improvement is needed. In order to expand physical training, Martinescu-Bdlan proposed a martial arts training method and also provided an effective method for athletes to warm up or perform other exercises [4]. However, this method involved many complex actions, which led to a high threshold and could not be widely promoted. Sulyma introduced modern technology and proposed that endogenous hypoxic respiration technology had a good application effect in the physical training of qualified hockey players [5]. However, the sports field of this study was too unpopular, and this technology had not been applied in other fields, so the research results are not very informative.

The article "Application of Biomechanics Based on Intelligent Technology and Big Data in Physical Fitness Training of Athletes" was retracted in 2023. Reasons: unreliable results or conclusions; concerns about the data; concerns about the peer review; concerns about the citations.

The development of technology has made physical training a better and safer way to achieve better results than before. Among them, intelligent big data and biomechanics are good research methods. He proposed an ensemble framework that enabled dynamic orchestration of network, cache, and computing resources—a novel deep reinforcement learning method for big data [6]. This method is used in many fields because of its good effect on data analysis, but the accuracy of this method needs to be improved. The big data computing method proposed by Xue can analyze key data in many different fields and solve the problem of the high computational complexity of the compressed sensing algorithm [7]. However, this method still lacks effective examples, resulting in a lack of practical significance. In addition to intelligent big data, biomechanics is also regarded as one of the good methods for physical training research. Retrouvey first applied biomechanics to orthodontics, which was ergonomic and promoted the development of biomechanics [8]. Although his research is innovative, it is more theoretical than practical. Guerra proposed an application in the biomechanics of human standing, in which unknown input observers were designed as tools for calculating joint torque and velocity [9]. This research has effectively promoted the development of biomechanics in various aspects of human training, but further research is needed if it is applied to other fields.

## 3. Methods for Improving Physical Fitness of Athletes, Taking Sprint Training as an Example

This section mainly introduces the methods of improving physical fitness training of athletes, mainly starting with the sport of sprinting. Before carrying out specific improvement behaviors, relevant data collection and analysis must be carried out first. By combining intelligent big data technology, monitoring, analyzing, evaluating, and feeding back the relevant data such as exercise intensity or exercise frequency of athletes' physical training, a comprehensive digital training system is established, and then a more scientific and reasonable training program is designed to make physical training move towards digital and intelligent development [10, 11]. Digital technology is used to process relevant data such as biochemical indicators, load intensity, and load amount in athletes' training. Through monitoring, analysis, evaluation, and feedback of relevant data, the numerical range related to the “fatigue coefficient” can be obtained and then effectively reduce the injury probability of athletes and increase sports life [12, 13].  Figure 1 shows the process of data collection, analysis, and application of athletes' physical training series.

The article "Application of Biomechanics Based on Intelligent Technology and Big Data in Physical Fitness Training of Athletes" was retracted in 2023. Reasons: unreliable results or conclusions; concerns about the data; concerns about the peer review; concerns about the citations.

### 3.1. Collation Process of Athletes' Physical Fitness Data under Intelligent Big Data

The source of this data collection is 21 sprinters. 7 were from the Tsinghua sprint team and 14 were from the Shanghai Institute of Physical Education sprint team. The Tsinghua sprint team has always been in the leading position in China's sprint and has achieved world-renowned results in major competitions in various places [14]. The sprint team of the Shanghai Institute of Physical Education has also achieved great results in major competitions around the world. The effective subjects of the Tsinghua sprint team included 4 athletes at the athlete level and 3 athletes at the first level, whereas the sprint team of Shanghai Institute of Physical Education consisted of 3 first-level sprinters and 11 second-level athletes.

First of all, it is necessary to carry out mathematical statistics. Based on sorting and summarizing the relevant index data, including biochemical indicators, load intensity, load, etc, the specific data of each training process of the athletes are monitored, and the relevant data are analyzed by the gray relational analysis method and the progressive scoring method, and the SPSS19.0 data processing software is used to determine each index. Finally, the physical fitness index evaluation and monitoring system is established, and the feedback system is improved. The related function arrangement in the Excel table processor is used to analyze the monitoring data.

The article "Application of Biomechanics Based on Intelligent Technology and Big Data in Physical Fitness Training of Athletes" was retracted in 2023. Reasons: unreliable results or conclusions; concerns about the data; concerns about the peer review; concerns about the citations.

In the actual analysis of the abovementioned relevant index data, the whole analysis process becomes more complicated due to the existence of certain connections between the variables. Therefore, it is necessary to use factor analysis to process the obtained data, simplify the analysis process, and make the analysis results simpler and clearer [15]. The specific process is as follows: First, the data that are determined to participate in factor analysis are sorted, then the R-type matrix of the relevant data is obtained, and the KMO moderate test and Bartlett's sphericity test are carried out on it. Next, the principal component analysis method is used to extract the specified factors to rotate the factor loading matrix with maximum variance, and, finally, the rotated factor scores are calculated and the factors are named.

Next, the gray correlation analysis method is used to analyze the correlation coefficient and weight value of each physical fitness index to verify the validity of the index screening results and factor analysis results and combine the particularity and the universality. The gray system theory believes that the world is not black and white, and different perspectives have different views on the “gray system.” From a mathematical point of view, this is a new “approximation” approach [16]. The approach here refers to the further measurement of the correlation degree. The specific operation process and calculation formula are as follows:

The generating function *X*_0_ and sub-function *X*_1_, *X*_2_, *X*_3_, *X*_*n*_ are determined, and *X*_*i*(*k*)_ is obtained as follows:

(1) $$\begin{array}{c} X_{i\left(k\right)}=\frac{Xi\left(k\right)}{X}. \end{array}$$

The absolute value of the difference (sequence) of the sub-function and the generating function is obtained as follows:

(2) $$\begin{array}{c} \Delta i\left(k\right)=\left|X_{0}\left(k\right)-X_{i}\left(k\right)\right|. \end{array}$$

Next, the difference between the two extremes is found, the purpose of finding the difference between the two extremes is to better find the correlation degree next:

(3) $$\begin{array}{c} \Delta \max=\max\left|X_{0}\left(k\right)-X_{i}\left(k\right)\right|,\\ \Delta \min=\min\left|X_{0}\left(k\right)-X_{i}\left(k\right)\right|. \end{array}$$

The correlation coefficient between the reference sequence (the generating function sequence) and the comparison sequence (the sub-function sequence) is as follows:

(4) $$\begin{array}{c} \varepsilon \left(k\right)=\frac{\Delta \min+\rho \Delta \max}{\Delta i\left(k\right)+\rho \Delta \max}, \end{array}$$

where *ρ* is the resolution coefficient, which is generally taken as 0.5, and the correlation degree is

(5) $$\begin{array}{c} r_{i}=\frac{1}{n}\sum \frac{n}{i=1}\varepsilon \left(k\right). \end{array}$$

After the correlation degree is obtained, the next step is to calculate the weight, which is given as follows:

(6) $$\begin{array}{c} \beta_{i}=\frac{ri}{\sum n/i=1ri}. \end{array}$$

There is an obvious feature of sports, that is, the higher the level of exercise, the more difficult it is to increase the performance by 1 unit. The same is true of the athletes' physical fitness level. The establishment of the athlete's physical fitness scoring method by the method of progressive scoring can make the physical fitness scoring more scientific and effective [17]. The specific process is as follows: First, the starting point and the full point are specified, the purpose of specifying the starting point and the full point is to have a minimum value and a maximum value during operation; and second, the progressive scoring formula is established. The progressive scoring formula is as follows:

(7) $$\begin{array}{c} y=kd^{2}-Z. \end{array}$$

It can be deduced from the cumulative scoring formula:

(8) $$\begin{array}{c} D=\sqrt{\frac{y}{1.56}}, \end{array}$$

(9) $$\begin{array}{c} x=\left(\sqrt{\frac{y}{1.56}}-5\right)\sigma +\bar{X}. \end{array}$$

Finally, according to formulas (8) and (9), when *y*=1,2,3,4,5,…, 10, the corresponding value of *X*_1_, *X*_2_, *X*_3_, *X*_4_,…, *X*_10_ can be obtained.

The article "Application of Biomechanics Based on Intelligent Technology and Big Data in Physical Fitness Training of Athletes" was retracted in 2023. Reasons: unreliable results or conclusions; concerns about the data; concerns about the peer review; concerns about the citations.

With the improvement of the physical fitness level of athletes, the growth rate of various physical fitness gradually decreases, and athletes' pursuit of physical fitness gradually fades. Long-term accumulation may lead to physical shortcomings in athletes, gradually increasing the distance between them and elite athletes, which is not conducive to the long-term development of athletes [18]. In view of the above situation, the comprehensive evaluation standard of physical fitness is used to comprehensively evaluate the athletes, so that the overall physical fitness level of the athletes can be steadily improved, and the concept of reflecting the overall level by individual quality is rejected. The specific steps for establishing a comprehensive level of physical fitness evaluation standard are: First, corresponding to the sprinter's scoring standard, the athletes' various physical qualities are “digitized,” and the specific scores of the athletes' 10 indicators *X*_1_, *X*_2_, *X*_3_,…, *X*_10_ are obtained. Second, the average fitness score of ${\bar{X}}_{a},{\bar{X}}_{b},{\bar{X}}_{c},\ldots ,{\bar{X}}_{n}$ for each athlete is calculated.

(10) $$\begin{array}{c} \bar{X}a=\frac{Xa1+Xa2+Xa3+\cdots Xa10}{10}. \end{array}$$

Then, the mean and standard deviation of ${\bar{X}}_{a},{\bar{X}}_{b},{\bar{X}}_{c},\ldots ,{\bar{X}}_{m}$ are obtained. Finally, the evaluation grades are divided in the form of the mean plus or minus the standard deviation, and it is stipulated that the first grade is excellent and the third grade is poor. The calculation formula of the mean and the standard deviation is as follows:

(11) $$\begin{array}{c} {\bar{X}}_{\text{score}}=\frac{{\bar{X}}_{a},{\bar{X}}_{b},{\bar{X}}_{c},\ldots ,{\bar{X}}_{m}}{n},\\ \sigma_{\text{score}}=\sqrt{\frac{\sum \left(xi-{\bar{x}}_{\text{score}}\right)}{n-1}}. \end{array}$$

In the process of sports training, balance is an important indicator to evaluate the coordinated development of various physical qualities of athletes, and the impact of various physical qualities on special performance is very important. When a certain physical fitness value of an athlete deviates from the normal range, corresponding measures should be taken in time to guide the long-term development of the athlete [19]. The balance of physical fitness in this study is denoted by ${\bar{X}}_{\Delta x}+\sigma_{\Delta x}$, in which:

(12) $$\begin{array}{c} {\bar{X}}_{\Delta x}=\frac{\Delta Xa+\Delta Xb+\Delta Xc+\cdots +\Delta Xn}{n},\\ \sigma_{\Delta x}=\sqrt{\frac{\sum n/i=a\left(xi-\bar{x}\Delta x\right)2}{n-1}},\\ \Delta xa=xa_{\max}-xa_{\min}. \end{array}$$

Finally, it is necessary to analyze the combination level of physical fitness, which refers to the degree of combination of physical fitness and technology. It is generally believed that the higher the level of physical fitness, the greater the potential for improving special performance. The relationship between physical fitness and technology is mainly different from person to person, and different athletes have different special combination abilities [20]. Therefore, based on the difference between the comprehensive level of athlete's physical fitness and the level of special performance, the level of integration of athletes' physical fitness and technique is evaluated. The combination of physical fitness is represented by *γ*:

(13) $$\begin{array}{c} \gamma_{a}={\bar{X}}_{a}-Y_{a}, \end{array}$$

where ${\bar{X}}_{a}$ is the average score of the 10 indicators of the athlete, and *Y*_*a*_ is the special score corresponding to the athlete. The closer the value of *γ* is to zero, the higher the degree of binding between the two, and vice versa. According to the normal distribution principle $\bar{\gamma }\pm \sigma_{\gamma }$, the specific formulas are as follows:

(14) $$\begin{array}{c} \bar{\gamma }=\frac{\gamma a+\gamma b+\gamma c+\gamma n}{n},\\ \sigma_{\gamma }=\sqrt{\frac{\gamma_{i}-\gamma -2}{n-i}}. \end{array}$$

The article "Application of Biomechanics Based on Intelligent Technology and Big Data in Physical Fitness Training of Athletes" was retracted in 2023. Reasons: unreliable results or conclusions; concerns about the data; concerns about the peer review; concerns about the citations.

### 3.2. Calculation of the Trainee's Movement from the Perspective of Biomechanics

In order to further improve the performance of athletes in sprinting and reduce the possibility of injury to athletes, this section uses Visual to model and calculate the human body, which is convenient for summarizing the exercise postures and movements of the best training mode after data collection to extract the correct movement posture and angle to provide reference for athletes' physical training. The human body modeling calculation of the software needs to capture the motion form of the human body.

First, the kinematics, kinetics, and EMG data of sprint were collected by Vicon infrared motion capture system, Kistler force plate, and Delsys wireless EMG acquisition system, respectively. Two days before the official collection, a sports biomechanics test base station was established in the indoor track and field gym. Subjects wore professional sprint sportswear and running shoes. Before training begins, the athlete warmed up fully for 15 minutes as usual. Warm-up exercises included static muscle stretches such as leg presses, dynamic muscle stretches such as high leg raises, jogging, and accelerated running. Then the formal sprint training began.  Figure 2 is a schematic diagram of the division of the sprint cycle of the athlete training to be recorded.

According to Figure 2, sprinting is divided into stages such as acceleration and landing, including ground support and reaction, and the human body vacates and accelerates. The Vicon processing software is used to grab the marker points captured by the motion capture system during acquisition. Grab points need to collect complete actions to be effective. The time length of the grab point is a complete support period and swing period, and 5 frames are added before the support period touches the ground and after the swing period leaves the ground, which is used for the calculation of the interaction dynamics of the sprint.

The sprint motion files that have been captured and intercepted are exported as .C3D files and imported into Visual 3D software for filtering processing and building a human model to calculate the center of gravity of the body. The .C3D file of the filtered sprint motion is saved for subsequent link interaction dynamics calculations of the lower extremity joints [21]. In addition, the .C3D file of the static calibration action collected during the experiment is exported from the Vicon data processing software, and it is ensured that all 53 marker points are not omitted before exporting. The static action .C3D file is imported into Visual 3D software, and the human body model is established based on the 15-link human body model to calculate the position of the center of gravity of the body [22–24]. The anthropometric data such as joint mass and moment of inertia required for building a human body model are the default values of V3D.  Figure 3 is a schematic diagram of the calculation of joint angles for sprint training.

The article "Application of Biomechanics Based on Intelligent Technology and Big Data in Physical Fitness Training of Athletes" was retracted in 2023. Reasons: unreliable results or conclusions; concerns about the data; concerns about the peer review; concerns about the citations.

According to Figure 3, after the human body model is established, the trajectory and speed of the center of gravity of a sprint gait cycle are calculated. The specific operation process is as follows: First, the .C3D file for the static calibration motion of the athlete in Visual 3D is imported. Second, the built mannequin file .mdh is applied to the static calibration action, and the height and weight of the athlete are modified individually. Then the .C3D file of the sprint motion that has been patched and intercepted before is imported, and the static calibration motion that has been modeled is applied to the sprint motion [25–27]. Finally, Visual 3D's built-in Pipeline data processing program is used to calculate the center of gravity trajectory and obtain the center of gravity velocity by one derivation. The average speed of the center of gravity in the fore-and-aft direction over the entire gait cycle represents the sprint speed [28, 29].

## 4. Experiments on Improving Physical Fitness Training of Athletes from a Biomechanical PerspectiveTaking Sprint Training as an Example

In this experiment, 8 sprinters (second-level) of Shanghai Institute of Physical Education were selected as the experimental objects, the experimental site is located in the gymnasium of Shanghai Institute of Physical Education, and the MotionPro X camera and its acquisition software were used to collect the raw data of running kinematics on the way (40 m from the start). The SBCAS kinematics processing software was used for processing and analysis, and the final data results were subjected to repeated measures analysis of variance using SPSS18.0 statistical software, and paired sample test was used for multiple comparisons. The venue used for the experiment was the indoor track and field of the Shanghai Institute of Physical Education, and the starting line, the ending line, and the viewing range were marked with a ruler and a tapered marker. The camera was placed 40 meters away from the starting line, and its main optical axis was 35 meters away. The camera height is 1.2 meters, the field width is 8 meters, and the high-speed camera sampling frequency is 100 HZ. The schematic diagram of the experimental site is shown in Figure 4.

### 4.1. Experiments on Biomechanical Characteristics of Athletes in the Acceleration Stage of Sprinting

In this section, the link interaction dynamics method was used to calculate the dynamic data of the lower limb joints, and this method attempted to explore whether there was a difference in the interaction between the active muscle torque and other passive torques during the acceleration phase and the maximum speed phase of the sprint. First, the athletes were subjected to sprint acceleration training, and the results of the hip and knee joint movements of the athletes were recorded during the swing phase of the acceleration phase. The force component curves of the hip and knee joints in the swing phase of the acceleration phase are obtained in Figure 5.

The article "Application of Biomechanics Based on Intelligent Technology and Big Data in Physical Fitness Training of Athletes" was retracted in 2023. Reasons: unreliable results or conclusions; concerns about the data; concerns about the peer review; concerns about the citations.

As shown in Figure 5, for the swing phase of the acceleration phase, since there was no ground reaction force acting on the lower limbs, there was no contact moment component for the lower limb joints. In the hip joint, it was mainly inertia moment and muscle moment. During the period from about landing to 50% swing, the muscle moment flexed the hip against the inertia moment. During the period of about 50% swing, until the foot left the ground, the muscle moment was always the hip extension moment, and the inertia moment was always the hip flexion moment. For the knee joint, at about 30% of the stance, the net torque was converted to the knee extension torque. At about 60% stance, the net moment turned back to the knee flexion moment. During the period from landing to about 60% support, the net moment and inertia moment were in the same direction, and the muscle moment was opposite to these two moments. This indicated that the moment of inertia completed the flexion and extension of the knee successively, and during this process, the confrontation between the muscle moment and the moment of inertia played a role in regulating the movement.

In the initial stage of support, especially in the maximum speed stage, there was a large contact moment between the hip joint and the knee joint; in the final stage of swing, there was a large moment of inertia. Active muscle torque opposed these two passive torques at the beginning of support and at the end of swing, respectively [30]. After understanding the relationship of the torque components, the test athletes were further accelerated, and the camera system was used to obtain the comparison of the lower limb muscle amplitudes of the athletes during the acceleration phase and the maximum speed phase, as shown in Figure 6.

According to Figure 6, in the forward swing phase, the athlete folded the lower limbs and swung the lower limbs forward to the highest point. The acceleration phase and the maximum velocity phase had a significant difference in the activation of the anterior thigh muscle-rectus femoris (*P*=0.037), the vastus medialis (*P*=0.027), and the posterior calf muscle-lateral gastrocnemius head (*P*=0.031). The degree of muscle activation during the maximum velocity phase was significantly greater than that during the acceleration phase. There was no significant difference between the two sprint stages in the activation of other muscles [31]. During the backswing phase, the athlete swung the lower body back while extending the knee in preparation for landing. There were significant differences in the activation degree of the lateral gastrocnemius head (*P*=0.027), biceps femoris (*P*=0.009), and vastus medialis (*P*=0.041) between the acceleration phase and the maximum velocity phase. The degree of muscle activation during the maximum velocity phase was significantly greater than that during the acceleration phase. The activation of the biceps femoris muscle, the posterior thigh muscle, differed the most between the two sprint stages (*P*=0.009). In the degree of activation of other muscles, there was no significant difference between the two sprint stages.

The article "Application of Biomechanics Based on Intelligent Technology and Big Data in Physical Fitness Training of Athletes" was retracted in 2023. Reasons: unreliable results or conclusions; concerns about the data; concerns about the peer review; concerns about the citations.

For the ground reaction force factor, the results of the experiments in this section reflected an interesting phenomenon: The braking force in the acceleration stage was significantly smaller than that in the maximum speed stage (−0.67 ± 0.25 vs. −1.30 ± 0.20), while there was no significant difference between the two propulsion stages (0.90 ± 0.11 vs. 0.88 ± 0.13). This showed that in terms of ground reaction force, compared with the maximum speed stage of sprinting, the increase in the body's center of gravity speed in the acceleration phase did not depend on greater propulsion but on a smaller braking force.

### 4.2. Experiments on the Physical Performance of Athletes by Applying Resistance Conditions

After the experiments on the link interaction dynamics and joint torque were completed, the content of this section was the biomechanical changes of the athletes' sprinting technique under the conditions of applying different resistances and assists so as to understand under which conditions the athletes could achieve the best training effect. The experiments in this section tested the physical performance of athletes under resistance loads of 0% BW, 10.6% BW, 14.1% BW, and 16.2% BW.

First, the acquired image data were obtained on the SBCAA and CAI SYSTEM-SBCAS kinematics processing software to obtain the *X* and *Y* coordinates of 18 key points. Through the 18 key points, the human body was defined with 14 links. The position coordinates of the total center of gravity of the human body were obtained by using the German human inertial parameters. The experimental data were expressed as mean ± table standard deviation (*x* ± SD).  Table 1 is the gait index of the experiment in this section.

The article "Application of Biomechanics Based on Intelligent Technology and Big Data in Physical Fitness Training of Athletes" was retracted in 2023. Reasons: unreliable results or conclusions; concerns about the data; concerns about the peer review; concerns about the citations.

As shown in Table 1, the significant level of gait-related indicators was *α* = 0.008. The sprint acceleration stage and the maximum speed stage had significant differences in running speed, support period, and stride length, while gait cycle duration, stride frequency, and swing period had no significant differences. The *P* values of the gait cycle duration and stride frequency were both less than 0.05, but since the above six gait indicators belonged to the same data, there might be correlations between them, which would affect the statistical results. To avoid this effect, the Bonferroni-adjusted significance level was *α* = 0.008, resulting in no statistically significant difference between the gait cycle duration and stride frequency and between the acceleration phase and the maximum speed phase. Next, the time indicators of the ground reaction force in the sprint acceleration phase and the maximum speed phase of the experiment in this section were introduced, as shown in Table 2.

According to Table 2, the significant level of the ground reaction force index was *α* = 0.004. When *P* < 0.004, there was a significant difference in the ground reaction force index between the two stages of sprinting. The sprint support period was divided into a braking period and a propulsion period according to the direction of the ground reaction force. After the sprint hits the ground, there was a braking period followed by a propulsion period. After introducing the above environment and indicators, the resistance instrument was fixed for the exercise, and then 3 test runs were carried out. The resistance test was conducted; the test resistance was standardized according to the weight of the athletes; the test resistance was randomly selected; and the resistance load was set as 0% BW, 10% BW, 15% BW, and 20% BW. 3 times successful data were collected.

The experimental preset values of the resistance value were 0% BW, 10% BW, 15% BW, and 20% BW for the first time and 0% BW, 10.6% BW, 14.1% BW, and 16.2% BW for the second time. Through the study of the data, it was found that with the increase of the load, the speed would continue to decrease, and the results are shown in Table 3.

According to Table 3, the average velocity of the center of gravity of the athletes (*n* = 8) was 9.33 ± 0.34 m/s when the resistance load was 0% BW. When the load increased to 10.6% BW, the average velocity of the center of gravity was 8.09 ± 0.21 m/s and the velocity decreased by 4.6%. When the load increased to 14.1% BW, the average velocity of the center of gravity was 7.08 ± 0.51 m/s and the velocity decreased by 24.1%. When the load increased to 16.2% BW, the average velocity of the center of gravity was 6.73 ± 0.35 m/s and the velocity decreased by 27.9%. Compared with the center of gravity velocity when the resistance load was 10.6% BW, 14.1% BW, and 16.2% BW, the *P* value was less than 0.01, which was very significant.

The article "Application of Biomechanics Based on Intelligent Technology and Big Data in Physical Fitness Training of Athletes" was retracted in 2023. Reasons: unreliable results or conclusions; concerns about the data; concerns about the peer review; concerns about the citations.

According to the average speed of the athlete's center of gravity under resistance loads of 0% BW, 10.6% BW, 14.1% BW, and 16.2% BW, this article established a regression formula between the load and the average speed of the center of gravity at a distance of 40 meters from the starting line: Speed = 8.986–12.494 *∗* weight (%); the average speed of the athlete's center of gravity is shown in Table 4, and the linear regression formula is shown in Figure 7. Through this formula, the speed of control training can be determined according to the load.

The next step was to analyze the stride length and stride frequency after the test run. Through the analysis of the experimental step length and stride frequency results, with the increase of the resistance load, the stride length continued to decrease, and the stride frequency did not change significantly. The experimental results of step size and step frequency are shown in Figure 8.

It can be seen from Figure 8 that when the resistance load was 0% BW, the average step length of athletes (*n* = 8) was 2.22 ± 0.23 m. When the resistance load was 10.6% BW, the average step size was 1.97 ± 0.13 m and the average step size decreased by 11.3%, and there was a significant difference (*P*=0.03). When the resistance load was 14.1% BW, the average step size was 1.77 ± 0.18 m and the average step size decreased by 20.3%, with a significant difference (*P*=0.001). When the resistance load was 16.2% BW, the average step size was 1.64 ± 0.07 m and the average step size decreased by 26.1%, with a significant difference (*P*=0.001). Under different resistance loads, the stride frequency did not change significantly, the *P* values were all greater than 0.05, and there was no significant difference.

For sprinting, athletes try to maintain the balance of the body during running, neither making the body rotate back nor forward, if the resistance load is increased, an additional backspin torque will be generated [32]. In order to overcome the extra backspin torque generated by the athlete, the body posture will be adjusted accordingly, that is by moving the body's center of gravity forward, to overcome the extra torque generated by the pulling force.

Finally, the entire gait cycle time was 100% normalized, and an overall analysis of the hip, knee, ankle, and thigh link angles was performed throughout the cycle. There was a tendency for the hip angle to decrease as the resistance load increased. There was no significant change in the angles of the knee, ankle, and thigh joints with increasing resistance load. At the moment of kicking off the ground, the angle of the trunk link decreased with the increase of the resistance load.  Figure 9 shows the difference in the change of the joint angle when kicking off the ground during running.

The article "Application of Biomechanics Based on Intelligent Technology and Big Data in Physical Fitness Training of Athletes" was retracted in 2023. Reasons: unreliable results or conclusions; concerns about the data; concerns about the peer review; concerns about the citations.

It can be seen from Figure 9 that when the resistance load was 0% BW, the angle of the trunk link was −8.6 ± 4.0 degrees; when the resistance load was 10.6% BW, the trunk link angle was −17.8 ± 3.6*∗* degrees compared with the trunk link angle when the resistance load was 0% BW (*P*=0.011); when the resistance load was 14.1% BW, the trunk link angle was −25.2 ± 7.8 degrees and there was a significant difference (*P*=0.001) compared with the trunk link angle when the resistance load was 0% BW; and there was a significant difference (*P*=0.001) between the trunk link angle at a resistance load of 16.2% BW and a trunk link angle of −25.9 ± 3.4 degrees when the resistance load was 0% BW.

From the above experimental results, from the perspective of biomechanics, the athlete's ability to complete the acceleration of the body's center of gravity in the acceleration phase depended on the smaller horizontal braking force rather than the larger horizontal propulsion force. Therefore, based on the results of this study, it is of great significance to find an effective training method for the hamstrings and design corresponding training equipment to improve the effect of physical training and prevent the injury of the hamstrings. In addition, as the resistance load increases during the physical training process, the horizontal speed of the athlete decreases, so when training with the resistance load, the maximum speed should not exceed 90% of the maximum speed without resistance. The average horizontal maximum velocity decreases by approximately 9% when training under resistance load, and any increase in this range will have a negative effect on training performance.

## 5. Conclusions

This article collected and analyzed the data of athletes through intelligent big data, then studied the dynamics and kinematics of different stages of sprint training, and used the link interaction dynamics model to explore the motion control mechanism of different stages of the sprint. This article looks for the differences in the biomechanical indicators in the sprint stage so as to understand the difference in the ability requirements of athletes in different stages of sprint and provide a theoretical reference for improving the physical training mode and innovating training methods. Due to the limited length of the article, it cannot provide a clearer description of the method, and it is difficult to do more comparative experiments. The description of the method in this article is also too simplistic and lacks specific details. In the future, it is expected to use more detailed steps to conduct more experimental analysis so as to provide a better reference for the training of athletes.

The article "Application of Biomechanics Based on Intelligent Technology and Big Data in Physical Fitness Training of Athletes" was retracted in 2023. Reasons: unreliable results or conclusions; concerns about the data; concerns about the peer review; concerns about the citations.

## Figures and Tables

**Figure 1:** The collection and application process of physical training data.

**Figure 2:** Schematic diagram of cycle division for training sprints.

**Figure 3:** Schematic diagram of joint angle calculation for sprint training.

**Figure 4:** Schematic diagram of the experimental scene shooting.

**Figure 5:** Curves of moment components of hip joint and knee joint in the acceleration stage of sprint.

**Figure 6:** Comparison of lower limb muscle amplitudes during acceleration phase and maximum speed phase: (a) Pre-swing. (b) Post-swing.

**Figure 7:** Regression formula for speed and weight.

**Figure 8:** Comparison of step size and stride frequency experimental results.

**Figure 9:** Difference results of joint angle change when sprinting off the ground. (a) Body angle. (b) Off-ground angle.

**Table 1:** Gait indicators of one cycle in the acceleration phase of sprinting.

	Speed up phase	Maximum speed phase	Deduction	*P* value
Running speed (m/s)	7.85 ± 0.61	9.35 ± 0.58	−1.50 ± 0.48	<0.001
Gait cycle duration	0.51 ± 0.05	0.48 ± 0.04	0.03 ± 0.03	0.026
Cadence	1.99 ± 0.19	2.06 ± 0.15	−0.07 ± 0.16	0.037
Length of support period	0.145 ± 0.014	0.128 ± 0.009	0.017 ± 0.012	<0.001
Swing period duration	0.363 ± 0.046	0.359 ± 0.035	0.004 ± 0.034	0.564
Step size	3.98 ± 0.27	4.50 ± 0.32	-0.52 ± 0.20	<0.001

**Table 2:** Time index of ground reaction force during the sprint acceleration phase.

	Speed up phase	Maximum speed phase	Deduction	*P* value
Braking period duration	32.2 ± 8.4	43.1 ± 3.2	−10.9 ± 8.2	<0.001
Propeller duration	67.8 ± 18.4	56.9 ± 3.2	−10.9 ± 8.2	<0.001
Peak braking moment	9.9 ± 4.8	10.0 ± 1.8	−0.1 ± 4.6	0.847
Peak propulsion moment	72.5 ± 3.5	72.7 ± 3.5	−0.2 ± 3.9	0.822
Vertical force peak time	37.6 ± 10.9	31.2 ± 1.8	6.4 ± 6.1	0.001

**Table 3:** Comparison of preset values and measured values.

Default value 1	0% BW	10% BW	15% BW	20% BW
Measured value 1	0% BW	10.6% BW	14.1% BW	16.2% BW
Default value 2	0.1% BW	11% BW	15% BW	17% BW
Measured value 2	0.1% BW	11.4% BW	15.3% BW	17.2% BW

**Table 4:** Average center of gravity velocity of athletes.

Load (% BW)	0% BW	10.6% BW	14.1% BW	16.2% BW
Average speed	9.34 ± 0.34	8.09 ± 0.21	7.08 ± 0.51	6.73 ± 0.35
Average speed	10.21 ± 0.31	9.21 ± 0.29	7.98 ± 0.87	7.15 ± 0.65
Average speed	10.06 ± 0.45	9.73 ± 0.39	8.25 ± 0.99	8.01 ± 0.36

The article "Application of Biomechanics Based on Intelligent Technology and Big Data in Physical Fitness Training of Athletes" was retracted in 2023. Reasons: unreliable results or conclusions; concerns about the data; concerns about the peer review; concerns about the citations.

## Data Availability

The data that support the findings of this study are available from the corresponding author upon reasonable request.
